# Factors influencing volatile fatty acids production from food wastes via anaerobic digestion

This article has been retracted.

**DOI:** 10.1080/21655979.2019.1703544

**Published:** 2019-12-27

**Authors:** Lukitawesa, Regina J. Patinvoh, Ria Millati, Ilona Sárvári-Horváth, Mohammad J. Taherzadeh

**Affiliations:** a Swedish Centre for Resource Recovery, University of Borås, Borås, Sweden; b Department of Chemical and Polymer Engineering, Faculty of Engineering, Lagos State University, Lagos, Nigeria; c Department of Food and Agricultural Product Technology, Universitas Gadjah Mada, Yogyakarta, Indonesia

**Keywords:** Inoculum to substrate ratio, pH control, the inhibitor for methanogens, O_2_, inoculum acclimatization, VFA, anaerobic digestion

## Abstract

Volatile fatty acids (VFAs) are intermediate products in anaerobic digestion. The effect of substrate loading or inoculum to substrate ratio (ISR), the addition of methanogen inhibitor, O_2_ presence, control the reactor’s pH, and inoculum adaptation on the VFAs production from food waste through acidogenesis process was investigated in this study. Addition of 2-bromoethane sulfonic (BES) as methanogen inhibitor suppressed VFA consumption by methanogens at ISR 1:1. At higher substrate loading (ISR 1:3), methane production can be suppressed even without the addition of BES. However, at high substrate loading, controlling the pH during acidogenesis is important to achieve high VFAs yield. Acclimatization of inoculum is also one of the strategies to achieve high VFA yield. The highest VFAs yield obtained in this work was 0.8 g VFA/g VS _added_ at ISR 1:3, controlled pH at 6, with the presence of initial O_2_ (headspace unflushed).

## 1. Introduction

Globally, about 1.3 billion tons of food wastes (FW) are disposed of annually, which is expected to increase significantly due to population and economic growth [1]. FW is an easily degraded waste fraction with high carbon content. However, improper treatment of these types of wastes will generate leachate and greenhouse gases (GHG) as well as the loss of valuable energy content. According to the Directive 75/442/EEC of the Economic European Community [2], reuse and recycling are the most favored options of waste management after waste prevention. In this context, traditional direct disposal and treatment techniques, such as landfilling or incineration, which are currently widely applied for FW, are the least sustainable choices. Landfilling leads to several environmental issues, including leaching, greenhouse gas emission (i.e., methane), and odor production. Moreover, this practice has increased costs imposed by EU landfill directives, which will eventually limit its application [3].

Due to the high moisture content of FW, incineration is an energy-demanding and inefficient process that also causes air pollution. Two other common practices for FW treatment are aerobic composting and the production of animal feed [4,5]. These options involve FW valorization, but generating low value-added products in the case of compost and increasing the risks of disease propagation in the case of animal feed application. Thus, there is an urgent need to develop and optimize alternative technologies for FW valorization and recycling. In their study, Chen et al. [6] found a considerable increase in the number of publications dealing with FW in the last years, evidencing the growing need to find alternative treatments for FW. Anaerobic digestion (AD) of food wastes has been reported as an environmentally viable and cost-effective treatment method compared to landfilling, incineration, and composting [7–9]. Commonly in the anaerobic digestion process has the main ultimate product is biogas. However, biogas production has its economic challenge, and without incentives, biogas cannot compete with conventional fossil fuels [10,11].

Volatile fatty acids are essential intermediates produced in the acidogenesis and acetogenesis step when organic materials are degraded by anaerobic digestion. VFAs have various applications, such as used as the carbon source in biological denitrification [12], production of biodiesel [13], generation of electricity through microbial fuel cells [14], and synthesis of complex polymers [14]. In recent years, VFAs and their derivatives have been widely used in food, textile, pharmaceutical, leather, and plastic industries [15]. Besides VFAs, during acidogenesis hydrogen gas is also produced [16], which is known as an ideal, clean, and renewable energy due to its combustion product that is only water [17]. In general, VFA production from waste can be achieved through the first two steps in an anaerobic digestion process, i.e., hydrolysis followed by acidogenesis (the latter also known as acidogenic fermentation [18] or dark fermentation [19]). During hydrolysis, complex organic polymers in waste are broken down into simpler organic monomers by enzymes excreted by hydrolytic microorganisms. Then, acidogens ferment these monomers into mainly VFAs, such as acetic, propionic, and butyric acids.

The production of VFAs from food wastes requires optimal conditions aiming to enhance the digestion process for industrial feasibility. The total concentration and type of VFAs produced depend on the substrate composition, operational parameters, available microbial community, type of reactor, and the process design [20–23]. In order to produce VFAs from food wastes through anaerobic digestion, the last step, the methane production, has to be inhibited. Some studies have shown that 2-bromoethane sulfonic (BES) has the ability to inhibit the activity of the methanogens [24,25]; having an optimum concentration of around 50 Mm for complete inhibition [25]. In another study, it has been reported that the use of 1 µmol/mL of BES could reduce the activity of methanogens by 60%, leading to an increased acetate accumulation [26].

Optimum pH between 4 and 5 was used in some studies with mixed cultures. Other researchers have reported pH 6 under varying conditions using activated sludge [23,27]. Alkaline conditions with pH around 9 to 10 have also been reported [28], but this is not suitable for industrial applications since it will increase the costs and the environmental impact of the whole process. Various researchers have reported total VFAs production from food waste around 7 g/L to 37.1 g/L at varying conditions with and without pretreatment of the food wastes [22,27,29,30]. However, those studies usually only cover one or two factors (pH, ISR, methanogen inhibitors, and O_2_ presence) at the same time, while these factors can have some synergistic effects. Therefore, it is crucial to consider the effects of these factors simultaneously on the production of VFAs, to see, for example, the interactive effects of pH and inoculum to substrate ratio (ISR) on VFA production [31,32]. The interaction effect between factors can be favorable or not favorable for VFA production.

Therefore, the aim of this study was to investigate the individual and interaction effect of factors such as pH (uncontrolled and controlled), inoculum to substrate ratio (ISR) and the addition of inhibitor for methanogens on concentration and composition of VFAs produced from food wastes in order to determine the optimum operating conditions to be used in future continuous digestion processes.

## 2. Materials and method

### 2.1. Substrate and inoculum

The composition food wastes usually vary, and as such, the substrate was prepared according to a previous work [33], based on average compositional analysis of food waste in European Union (EU), to reduce experimental bias; consisting of 79% fruits and vegetables, 5% pasta and rice, 6% bread and bakery, 8% meat and fish, 2% dairy product (on the basis of wet weight). These ingredients were purchased from a local supermarket in Borås, Sweden. The food items were cut into pieces and then homogenized using countertop blender thereafter characterized, weighted, and stored in plastic containers at −20°C to prevent biodegradation until further use. The chemical characteristics of substrate are presented in Table 1.

**Table 1.** Characteristics of food waste in this study.

Parameters	Percentage
TS (%)	17.8
VS (% db)	95.8
Protein (% db)	21.3
Lipid (% db)	3.3
Ash (% db)	4.2
Crude fiber (% db)	2.5
Pectin (% db)	3.7
Carbohydrate (by difference) (% db)	70.4
Total COD (g/L)	320
Soluble COD (g/L)	95
C/N	15.6
%TSS	8.7

Sludge used as inoculum was obtained from a digester treating excess sludge from a wastewater treatment plant and operating at mesophilic conditions (Vatten and Miljö I Väst AB, Varberg, Sweden). The inoculum was filtered through a 2 mm porosity sieve to remove undesired particles, after which it was acclimated for 5 days in an incubator at 37°C to be stabilized prior to use.

### 2.2. Effect of initial O_2_ presence, addition of inhibitor for methanogens, and ISR on the production of VFAs

The experiments were carried out in factorial design with three factors at two levels each meaning 2^3^ sets of assays. The reactors were set to an initial pH of 6 without pH control afterward. Serum glass bottles of 120 ml were used as reactors with a working volume of 55 ml and inoculum to substrate ratio (ISR) of 1:1 or 1:3 and with/without BES addition. The reactors were then closed tightly, and half of them were flushed with a gas mixture of 80% N_2_ and 20% CO_2_ for 2 min to obtain anaerobic conditions, while the other half were not flushed to obtain the effects of non-strict anaerobic conditions (with the presence of O_2_) used. Finally, all reactors were incubated in a water bath shaker at 37°C and 100 rpm an investigation period of 14 days. All experimental setups were carried out in duplicates. Samples were taken every second day (i.e., at 2, 4, 6, 8, 10, 12, and 14 days) for the analysis of VFAs and for compositional analysis of the gas produced. The variations in pH and oxidation/reduction potential (ORP) during the investigation were also determined.

### 2.3. Effect of controlled pH conditions and ISR on the production of VFAs

The experimental setup was designed on the bases of results obtained from the previous experiment mentioned above. Experiments were carried out at different pH of 4, 5 and 6 and at two different ISRs (1:1 and 1:3) without the addition of BES, which means there were six different setups investigated. All experimental setups were carried out in duplicate in 2-L CSTR or continuous stirred tank reactors (Bioprocess control AB, Sweden) with a working volume of 1.5 L and incubated in a water bath at 37°C with 100 rpm agitation. The pH in all reactors was controlled at every second day and adjusted to the initial values of 4, 5 and 6 using 5 M NaOH or 5 M HCl and there was no flushing with a gas mixture of 80% N_2_ and 20% CO_2_, neither at the beginning of the experiment nor during the adjustments of the pH. Samples (10 ml) were taken in every second day for the analysis of VFAs and ammonium nitrogen (NH_4_-N), as well as gas samples, were also taken for compositional analysis of the gas produced. Gas samples were taken from the headspace of each reactor using a 250-μl pressure-lock gas syringe (VICI, precious sampling Inc., USA).

### 2.4. Analytical methods

The moisture content, total solid (TS), volatile solids (VS), and volatile suspended solids (VSS) of substrates and inoculum were determined according to biomass analytical procedures [34]. Total Kjeldahl nitrogen (TKN) contents were measured using the Kjeldahl method, and the protein content was estimated by multiplying the TKN content with a factor of 6.25 [35]. Total carbon was obtained by correcting the total dry weight carbon value for the ash content [36,37]. Fat content was determined using the Soxhlet extraction procedure [38]. Samples from reactors were centrifuged (5 min at 20,000 × *g*), and supernatants were collected for the analyses of VFAs and NH_4_-N.

VFAs were measured using high-performance liquid chromatography (HPLC, Waters 2695, Waters Corporation, Milford, MA, USA) equipped with a biohydrogen-ion exchange column (Aminex HPX-87H, Bio-Rad, Hercules, CA, USA) operating at 60°C. For the determinations, an UV absorbance detector (Walters 2487, Waters Corporation Milford, MA, USA), operating at 210 nm wavelength was used in series with a refractive index (RI) detector (Waters 2414, Waters Corporation Milford, MA, USA) operating at 60°C. Prior to analysis, samples were first centrifuged at 20,000 × *g* for 10 min to exclude the natant from the analysis. The supernatant was then filtered using an HPLC certified syringe filter (GHP Acrodisc 13 mm with 0.2 μm GHP membrane) to remove remaining contaminant particles, which might hinder column separation. The NH_4_-N was measured using the Ammonium 100 test kit (Nanocolor, MACHEREY-NAGEL GmbH & Co. KG. Germany), and concentrations were determined using Nanocolor 500D Photometer (MACHEREY-NAGEL GmbH & Co. KG. Germany).

The total volume of gas produced from 2 L CSTR was measured by the tipping device in the Automatic Methane Potential Testing System (AMPTS, Bioprocess control AB, Lund, Sweden). The gas production, yield, and composition were determined based on a measurement using Gas Chromatography (Varian 450 GC, Palo Alto, CA, USA). A gas sample (100 μL) was withdrawn using a 250-μL gas-tight syringe equipped with a pressure lock (VICI, Baton Rouge, LA, USA). It was then injected and analyzed with Varian 450 Gas Chromatography. The GC was equipped with a Wall Coated Open Tubular (WCOT, J & W Scientific GS-Gas Pro, bonded silica-based 30 m × 0.32 mm, Agilent Technologies, Santa Clara, CA, USA) capillary column, a thermal conductivity detector (TCD, Varian, Palo Alto, CA, USA) and Galaxie Chromatography Data System Single Instrument as the data recording software (v.1.9, Varian, Walnut Creek, CA, USA). Nitrogen was chosen as the carrier gas with flow rates of 2.0 mL/min passing the column and of 30 mL/min passing the detector. An injection split ratio was set at 5 with an injector temperature of 75°C. Meanwhile, the oven, detector heater, and detector filament temperatures were set at 55°C, 120°C, and 200°C, respectively. To ascertain peak retention time and calculate gas production, pure methane (CH_4_), carbon dioxide (CO_2_), and hydrogen (H_2_) were used as the standard. The calculation was later done by comparing the peak area of the sample and the peak area of the standard, followed by conversion to the steady-state condition (273 K).

### 2.5. Experimental design and statistical analysis

A two-level three-factor full-factorial experiment design (2*^k^*) was carried out to investigate the effects of ISR, initial O_2_ presence, BES, and the interaction between effects toward VFA yield and methane production in the first experiment (for section 2.2 and 3.1). Meanwhile, the general multilevel full factorial design was carried out to investigate the effects of pH, ISR, and the interactions between two factors toward VFA yield and methane production (see Sections 2.3 and 3.2)). The experimental design for each experiment is presented in Tables 2 and 3. All experimental setups were carried out in duplicates.

**Table 2.** Factors considered in the two-level full factorial design in Section 3.1.

Factor	Low level (−1)	High level (+1)
Initial oxygen presence (%)	0	20 – 20.5
Inhibitor for methanogens: 2-bromoethanesulfonate (BES) (g/L)	0	2
Inoculum to substrate ratio (ISR)	1:1	1:3

**Table 3.** Factors considered in the general multilevel factorial design in Section 3.2.

Factor	Low level (−1)	Mid-level (0)	High level (+1)
Controlled pH	4	5	6
Inoculum to substrate ratio (ISR)	1:1	-	1:3

To evaluate the influence of those factors, an analysis of variance (ANOVA) for the general multilevel factorial design was performed. The means of the significantly different main effects were compared at p < 0.05. The statistical analysis was performed using Minitab 19.

## 3. Result and discussion

In order to evaluate the effects of different digestion conditions, i.e., inoculum to substrate ratio (ISR), the presence of initial O_2_, the presence of inhibitor during anaerobic digestion of food waste, four response parameters were investigated, i.e., the yield of VFAs, the amount of produced gas, the pH, and the ORP. Based on the results of this first assay, in the second experiment, the effects of just ISR together with the effects of different controlled pH values were investigated by following up the same response parameters as within the first assays.

### 3.1. Effect of initial O_2_ presence, the addition of inhibitor for methanogens, and ISR on the production of VFAs

The production of VFAs through a conventional anaerobic digestion process can be performed by stopping the degradation process at the acidification step, to promote VFA accumulation. In order to promote VFA accumulation, the digestion conditions should be adjusted to achieve unsuitable conditions for methanogens [39], as methanogens are VFA consumers. Inhibition of methanogens can be performed by several different ways, i.e., by adjusting the pH, by adding a chemical inhibitor, such as 2-bromoethanesulfonate (BES) [25], or by the presence of O_2_ [39], as well as by increasing the substrate loading [39]. In this first experiment, the effects of inoculum to substrate ratio, the addition of BES, and the presence of initial O_2_ on the yield of VFAs obtained through batch digestion assays were determined and the results are shown in Figure 1. All of these assays were carried out at an initial pH of 6, and then the pH remained uncontrolled during an incubation period of 14 days.

**Figure 1.** (a)–(h) VFA yield during batch anaerobic digestion of food waste at pH 6 using different ISRs, with or without the addition of BES, and with or without the presence of initial O_2_. Ac: acetic acid, Pr: propionic acid, Bu: butyric acid, Iso-Bu: iso-butyric acid, Va: valeric acid, Iso-Va:iIso-valeric acid, Ca: caproic acid.

In general, reactors with ISR of 1:1 (Figure 1(a–d)) had higher yields of VFAs compared to those in reactors with ISR of 1:3 (Figure 1(e–h)). At ISR of 1:1, the addition of BES or the presence of initial O_2_ did not affect the VFA yield (Figure 1(a,b), *vs*. (c), (d), or 1(b), 1(d) *vs*. 1(a) 1(c), respectively), and the two dominant VFAs in all reactors were acetate and butyrate. However, the composition of VFAs was affected depending on the conditions, showing a substantially higher amount of caprionate, as the third main VFA component at conditions with BES and without O_2_ (Figure 1(a)) as well as at conditions without BES and with O_2_ (Figure 1(d)). The yield of VFA at ISR 1:1 after 12 days incubation was around 0.5–0.6 g VFA/g VS. The decrease of acetate concentration from 12th day to 14th day might be caused by acetate consumption by methanogens. The P-value of the addition of BES and the presence of initial O_2_ were larger than 0.05 (Table 5), indicating that those factors did not significantly affect VFA production at ISR 1:1. However, the presence of initial O_2_ might affect the VFA composition (Figure 1(c) *vs*. 1(d)) when the BES was not added.

**Table 5.** *P*-value of selected factors: inhibitor for methanogens (BES), initial oxygen presence (O_2_), and inoculum to substrate ratio (ISR).

	*P*-value for VFA yield	
Factors	**Day 12**	**Day 14**
**Main effects**		
Inhibitor for methanogens (BES)	0.848	0.128
Initial oxygen presence (O_2_)	0.891	0.330
Inoculum to substrate ratio (ISR)	0.004	0.000
**Two-way Interactions**		
BES*O_2_	0.783	0.867
BES*ISR	0.911	0.408
O_2_*ISR	0.859	0.118
**Three-way Interactions**		
BES*O_2_*ISR	0.783	0.537

Unlike methane production which is more susceptible with the exposure of O_2_, this result proves that VFA production is not significantly affected by the presence of O_2_ (p < 0.05, Table 5). In practical, this can be beneficial in industry when the reactor needs to be opened for maintenance. The addition of inhibitor for methanogens (BES) was also not significantly affect the VFA yield (p < 0.05, see Table 5). Therefore, the addition of BES might be unnecessary at high loading of substrate because usually the concentration of VFA itself is able to suppress the methanogens.

Meanwhile, the dominant VFAs in the reactor with ISR 1:3 were iso-valerate, butyrate, and acetate (Figure 1(c,d)). ISR was showing a significant effect toward VFA production in this experiment setup (p < 0.05), indicating that the VFA production at ISR 1:3 is significantly lower than that of ISR 1:1 (Figure 1(a–d) *vs*. Figure 1(e–h)).The substrate loading, in this case, ISR, can probably also affect the metabolic pathway of the mixed culture of microorganisms in anaerobic digestion. For instance, Jiang et al. [30] reported that the share of acetic acid concentration could decrease at low substrate loading compared to the share of the longer-chain acids, such as butyric and valeric acids.

Accumulated biogas yield, ammonium nitrogen, ORP, and pH during digestion were analyzed to evaluate the effect of different factors into an overall digestion of food waste. Ammonium nitrogen has been studied as an indicator of protein degradation in anaerobic digestion [40]. After the 12th day, the VFA yield decreased because there was methane production. This indicates that some parts of the VFA were consumed for methane production The addition of BES caused reduction in methane production at ISR 1:1. Without BES and in anaerobic condition (No O_2_), BES was able to suppress methane yield during digestion from 1.7 to 0.3 g mL methane/g VS. At the same ISR, the presence of O_2_ was also able to suppress methane yield from 1.7 to 0.8 mL methane/g VS even without the presence of BES (Table 4). However, the presence of initial O_2_ did not statistically have an effect on the methane yield. On the other hand, at ISR 1:3, addition of BES did not affect methane production. These results indicate the importance of BES and a small dose of O_2_ by not flushing the headspace with O_2_-free gas in low substrate loading (ISR 1:1). Suppressing methane production in anaerobic digestion is one strategy, which can be applied to achieve high VFA yield.

**Table 4.** Total VFA yield, ammonium nitrogen concentration, biogas yield, pH, and ORP during batch fermentation at different inoculum to substrate ratios, with and without the presence of BES, and with and without the presence of O_2._

	Total VFA yield		Ammonium nitrogen concentration (mg/L)	Gas yield a (mL/g VS) at day 12			ORP	pH
ISR/condition	Day 12	Day 14	Day 14	H_2_	CH_4_	CO_2_	Day 14	Day 14
1:1/BES. No O_2_	0.50	0.35	850	37.0	0.3	6.6	97.5	4.9
1:1/BES. O_2_	0.53	0.34	875	25.3	0.3	20.3	96.5	4.9
1:1/No BES. No O_2_	0.54	0.39	850	30.4	1.7	21.5	104.0	4.8
1:1/No BES. O_2_	0.52	0.35	825	25.5	0.8	11.1	100.0	4.9
1:3/BES. No O_2_	0.12	0.08	725	14.2	0.0	6.4	150.5	4.0
1:3/BES. O_2_	0.08	0.08	550	8.7	0.1	4.2	150.0	4.0
1:3/No BES. No O_2_	0.12	0.09	700	13.6	0.1	4.1	146.5	4.0
1:3/No BES. O_2_	0.08	0.09	700	11.1	0.1	5.8	147.5	4.0

The pH of the reactors with ISR 1:1 decreased from 6 into 4.6 by the 2nd day and bounced back 4.8–5 until the 14th day (Figure 2(a)). On the other hand, the pH of the reactor with ISR 1:3 decreased into 4 on the 2nd day and leveling off until the 14th day (Figure 2(b)). The presence of O_2_ and the addition of BES in both ISR did not affect the pH.

**Figure 2.** The pH (a and b) and ORP (c and d) of reactors at initial pH 6 (uncontrolled pH), different ISR, with and without the presence of BES, and with and without the presence of O_2._

### 3.2. Effect of different controlled pH on VFA production

The pH was shown to have an effect on the acidogenic fermentation type [41]. In order to investigate the effect of pH at different ISRs in the VFA production of food waste, three different controlled pH (4, 5, and 6) had been tested with two different ISRs (1:1 and 1:3). In the reactors with pH control, the pH was adjusted to 4, 5, and 6 every 2 days.

The pH control, in general, stabilizes the fermentation condition. The composition of VFA was different at different pH values. As the substrate loading (ISR) increased, the propionic acid also increased (Figure 3). At ISR 1:1, the yield of VFAs was higher compared to ISR 1:3. The pH 6 gave the highest VFA yield compared to the other pH values (4 and 5). The pH was reduced significantly on the 2nd day before returned back to the desired pH (Figure 4). At high substrate loading, i.e., ISR 1:3, the pH further reduced, indicating VFA production was higher than that of ISR 1:1. In a previous study [42], acidic pH values (pH 3–5) were not reported to be favorable for VFA production, while alkaline pH [43] was favorable for hydrolysis of complex organic matter [42]. The neutral pH (6–7) was beneficial for the acidogenesis and the overall VFAs production [42]. However, studies reporting the effect of pH in batch acidogenesis [21,23,42,44–46] were mostly only adjusting the initial pH without controlling throughout the digestion. pH (controlled) and ISR were significantly affecting VFA production (Table 7, p < 0.05).The present study shows that there is a two-factor significant interaction between the pH and ISR tested in this study (Table 7, pH*ISR).

**Figure 3.** (a)–)f) VFA yield during batch fermentation of food waste at different controlled pH and ISR. Ac: acetic acid, Pr: propionic acid, Bu: butyric acid, Iso-Bu: iso-butyric acid, Va: valeric acid, Iso-Va: iso-valeric acid, Ca: caproic acid.^Figure 1.^

**Figure 4.** pH (a and b) and ORP (c and d) during anaerobic digestion of food waste at different pH and ISRs.

**Table 7.** *P*-value for selected factors: pH and inoculum to substrate ratio (ISR).

	*P*-value for VFA yield	
Factors	**Day 12**	**Day 14**
**Main effects**		
pH	0.006	0
Inoculum to substrate ratio (ISR)	0.721	0
**Two-factor interactions**		
pH*ISR	0.050	0

A study by Lim et al. [29] reported that at pH 5.0, the acetic, butyric, and caproic acids were 18.2%, 18.4%, and 13.0% of the total VFA, respectively. The differences in the metabolic activities toward the production of different VFAs in undefined mixed culture systems, such as the one applied in our study, can also be ascribed to the microbial community structure enriched in the seeding inoculum due to the diversity of the bacteria and the available nutrients [47]. The production of acetic acid dominates when the pH is kept in the acidic region while operating around the neutral region has been reported to favor the production of longer-chain carboxylic acids [48].

Slightly acidic pH (6) shows to be better conditioned for VFA production. As shown in Table 6, the ammonia concentration at pH 6 was higher than at pH 4 and 5 at both ISRs. Higher ammonium nitrogen concentration most likely indicates that there was more protein degradation compared to the low ammonia concentration. In anaerobic digestion, the degradation of protein takes longer than carbohydrate degradation. It is most likely because of protein degradation is a complex multi-stage process, while carbohydrate degradation is a stepwise process [40]. Carbohydrate was degraded more efficiently than protein and degraded prior to protein during anaerobic sludge digestion [40]. Each protein compound can only be degraded by a specific type of protease, thus leading to various degradation rates of different kinds of protein compounds [40]. Degradation of protein indicates that the microbial community almost finishes degrading carbohydrates.

**Table 6.** Total VFA yield, ammonium nitrogen concentration and gas yield during anaerobic digestion of food waste at different controlled pH and ISR.

	Total VFA yield		Ammonium nitrogen concentration (mg/L)	Gas yield day 12 (mL/g VS)			pH	ORP
ISR/pH	Day 12	Day 14	Day 14	H_2_	CH_4_	CO_2_	Day 14	Day 14
1:1/pH 4	0.51	0.41	750	169.1	0.6	0.1	3.99	144.5
1:1/pH 5	0.58	0.58	800	122.9	3.3	0.4	4.98	88
1:1/pH 6	0.57	0.17	900	56.3	6.2	0.8	6.85	−19
1:3/pH 4	0.22	0.17	700	0.1	0.09	0.0	3.95	147
1:3/pH 5	0.58	0.48	875	70.0	0.4	0.1	4.96	89
F/1:3/pH 6	0.81	0.51	1225	51.3	0.4	0.0	5.96	32.5

The composition of VFA at pH 6 at lower substrate loading (ISR 1:1) was dominated by acetate, butyrate, and valerate. This result is in line with the metabolic pathway involved in the acidogenesis process (Figure 6), which was explained by Feng et al. [49]. Meanwhile, at higher substrate loading (ISR 1:3) at pH 6, acetate, butyrate and caproate dominates the VFA composition. The high production of butyric and caproic acids might be caused by high activity of the specific acid-producing bacteria [50,51]. Figure 7 shows the mass balance calculation for the VFA production at ISR 6 and pH-controlled at 6 (Figure 3 f at day 12) shows that 48 g VFA was produced from 60 g VS substrate and only a small amount of methane produced.

**Figure 5.** VFA yield during batch fermentation of food waste at initially adjusted to pH 6 but uncontrolled (a and b) and controlled at pH 6 through the experiments (c and d). The abbreviations of the individual acids are similar to Figure 2.

**Figure 6.** The metabolic pathway involved in acidogenesis process in anaerobic digestion. Adapted and modified from Feng et al. [49].

**Figure 7.** Mass balance illustration of the reactor with pH controlled at 6 and ISR 1:3.

Regarding gas production, at low substrate loading (ISR 1:1), the system produces methane with a yield of 6.2 mL/g VS at pH 6 and 3.3 mL/g VS at pH 5. At pH 6, the hydrogen yield was also lower than that of lower pH (4 and 5), which indicates that some of the hydrogens were consumed to produce methane by methanogens (Table 6). The decrease of VFA yield on the 12th day to 14th day was mainly caused by methane production.

On the other hand, at higher substrate loading (ISR 1:3), the methane was produced in a low amount with the yield of 0.4 mL/g VS at both pH 5 and 6 (Table 6). These results indicate that in order to suppress methane production to achieve high VFA production, the substrate should be loaded at high loading in order to suppress the growth of methanogenic community.

### 3.3. The importance of controlling pH on VFA production during digestion

pH is one of the crucial factors to achieve a high VFA yield. pH 6 has been shown to be a suitable condition to produce high yield VFA compared to lower pH (Figure 3). However, adjusting the initial pH, especially at high substrate loading (ISR 1:3), was not enough to achieve high VFA yield. As shown in Figure 5, initial pH adjustment at pH 6 without pH controlling (Figure 5(b)) during digestion give lower VFA yield (0.11 g VFA/g VS) compared to the reactor with pH control at 6 (Figure 5(d)) at 0.8 g VFA/g VS. On the other hand, controlling the pH was unnecessary at lower substrate loading (ISR 1:1) because it does not give a higher VFA yield (Figure 5(a,c)).

### 3.4. Effect of inoculum acclimatization on VFA production

In order to investigate the role of inoculum acclimatization, semi-continuous experiment with VFA extraction assisted by tubular membrane was carried out in 30 days. The first reactor (Figure 8(a)) was inoculated with the inoculum that had been fed with a high substrate loading for 14 days. Meanwhile, the second reactor was inoculated using fresh inoculum from a biogas reactor. As can be seen in Figure 8, acclimatization of inoculum was able to increase VFA production in the filtrate about 35 times from 0.45 g VFA/L into 16 g VFA/L. This result indicates that acclimatization of inoculum can shift the microbial community into VFA production instead of methane production. Another study [52] reported that the acclimatization process enriched the phylum *Firmicutes* (90%), followed by *Bacteroidetes* (12%) and *Cloacimonetes* (11%). The abundance of these phyla and their respective genera confirmed their preeminent role in hydrolysis, hydrogenogenic acidogenesis, and carboxylic chain elongation to produce hydrogen and C4–C7 fatty acids [52].

**Figure 8.** VFA concentration in the permeate of reactors with (a) and without (b) inoculum acclimatization during semi-continuous anaerobic digestion of food waste at organic loading rate (OLR) 1.0 g VS/L.day. Ac: acetic acid, Pr: propionic acid, Bu: butyric acid, Iso-Bu: iso-butyric acid, Va: valeric acid, Iso-Va: iso-valeric acid, Ca: caproic acid.

## 4. Conclusion

The presence of BES in the anaerobic digestion of food waste was able to suppress methane production at low substrate loading (ISR 1:1). At high substrate loading (ISR 1:3), the methane production was suppressed by itself. However, at high substrate loading, the pH has to be controlled during the batch anaerobic digestion. The presence of O_2_ was able to suppress methane production at low substrate loading (ISR 1:1) without affecting the VFA yield while the composition was slightly affected. Acclimatization of inoculum was also favorable to achieve a higher VFA yield. In practical application, controlling the pH is most likely the most important factor determining the VFA yield. Besides, as oxygen does not have a significant effect on the VFA yield, the presence of little oxygen or opening the reactor for maintenance does not harm the digestion process.

## Highlights

- Acidogenesis of food waste was better at controlled pH 6 at high substrate loading
- The methane production can be reduced by addition of inhibitor for methanogens
- The presence of initial O_2_ did not negatively impact the VFA yield
- Inoculum acclimatization can improve VFA production in anaerobic digestion
